The article "Psychological Characteristics and Health Behavior for Juvenile Delinquency Groups" was retracted in 2024. Reasons: signs of a paper mill; suspected computer-generated content; unreliable results or conclusions; lack of ethics approval or compliance.

# Psychological Characteristics and Health Behavior for Juvenile Delinquency Groups

**DOI:** 10.1155/2022/3684691

**Published:** 2022-08-02

**Authors:** Fangbin Song, Ruihua Li, Wei Wang, Shenyu Zhang

**Affiliations:** ^1^School of Design Art&Media, Nanjing University of Science and Technology, Nanjing, Jiangsu Province, 210094, China; ^2^School of Law, Southeast University, Nanjing, Jiangsu Province, 211189, China; ^3^School of Electronic Engineering, Jiangsu Ocean University, Lianyungang, Jiangsu Province, 222005, China; ^4^College of Liberal Art, Nanjing Normal University, Nanjing, Jiangsu Province, 210000, China

## Abstract

The related literature is studied to explore the psychological characteristics of juvenile delinquency groups and implement their psychological characteristics model for the intervention of health behavior. Drawing on the results of current literature research, the Youth Psychological Characteristics Crime Prevention Questionnaire (YPPQ) was compiled, which can be simply referred to as the Crime Prevention Questionnaire. The whole psychological characteristics of juvenile delinquency are analyzed by means of a questionnaire. Firstly, the YPPQ scores of different groups were compared, and a structured interview was conducted on the reasons for the crime of the problem youth group. Secondly, data analysis was carried out on the results of questionnaires and interviews, and the psychological characteristics of juvenile delinquency were summarized. A “mixed hierarchical intervention model” was proposed to intervene in the mental health behavior of juvenile delinquency groups, and corresponding intervention strategies were also proposed. The results reveal that through the questionnaire survey, the educational background of juvenile subjects was generally distributed in middle school, the number of juveniles with primary school education was less than 30% of the juvenile delinquency groups, the middle school education accounted for more than 60% of the juvenile delinquency groups, and the approximate age was about 18 years old. The largest number in each group were adolescents with secondary school education, indicating the importance of psychological education on crime prevention for adolescents in secondary school. By comparing the YPPQ test scores of different groups, the adolescent group has higher test scores than the juvenile delinquency groups in five of the dimensions. Through the comparative analysis of the YPPQ test results of the juvenile delinquency groups, the problem youth group, and the normal youth group, it is found that the YPPQ has high reliability and validity, so its detection and evaluation are highly feasible. By comparing the odds ratio (OR) of each question in the YPPQ test between the experimental group and the control group, it is found that the psychological characteristics of the experimental group are significantly affected by family, school, and even society. Finally, it proposes a “mixed hierarchical intervention model” for juvenile delinquency to intervene in health behaviors. The purpose is to provide some research ideas for the study of the psychological characteristics of juvenile delinquency groups and to put forward some suggestions for the prevention of juvenile delinquency and the intervention of health behavior.

The article "Psychological Characteristics and Health Behavior for Juvenile Delinquency Groups" was retracted in 2024. Reasons: signs of a paper mill; suspected computer-generated content; unreliable results or conclusions; lack of ethics approval or compliance.

## 1. Introduction

With the rapid expansion of China's economy and culture, the phenomenon of juvenile delinquency has gradually increased, and the education problems of juveniles have gradually been exposed, which has brought certain unsafe factors to the society, and even caused serious harm [1]. To prevent juvenile delinquency, the motives and psychological characteristics of juvenile delinquency must be understood. Therefore, the construction of the psychological characteristic model of juvenile delinquent groups is extremely important; in addition, it is particularly necessary to intervene in the mental health of the juvenile delinquent groups [2]. Juvenile delinquency is a behavior that deviates from social norms and moral norms and violates the law, which has aroused the concern of the whole society. Many studies show that the causes of different individuals who commit crimes are different [3]. Psychological characteristics are the most vital individual difference variables and the area that researchers pay the most attention to. Therefore, the predictive evaluation of the psychological characteristics of juvenile citizens' criminal tendency and the screening of people with psychological characteristics of juvenile delinquency is directly related to the stability of China's social order [4].

The research on the psychological characteristics of traditional juvenile delinquency groups has been difficult to meet the requirements of juvenile health cultivation. Some scholars have done some research on psychological quality testing. Guided by theories of mental health and the quality of Chinese adolescents' mental health, an online mental health assessment has an established system for primary and secondary schools, providing schools, teachers, and parents with a platform to better observe students' mental health. Relatively stable environmental factors influencing adolescent internalization problems are screened. Taking environmental factors as independent variables, the adjustment mechanism of adolescents' psychological traits affecting adolescents' internalization problems is explored, and ultimately, adolescents' psychological traits and the indicators of internalization problems are obtained [5]. Rodriguez-Ayllon et al. explored the relieving effects of different exercise intervention programs on adolescents' psychological stress and the characteristics of changes over time. Many students were used as subjects, and three kinds of intervention programs lasting 16 weeks were used to test the relieving effect on adolescents' psychological stress [6]. Lee et al. used a two-factor model to revise and test college students' psychological quality measurement tools [7]. The research literature found that there are few studies on the detection of adolescents' psychological quality, and the content urgently needs to be improved and supplemented. In the face of the group characteristics of juvenile delinquency, it is undeniable that the current law not only strengthens the protection of juveniles but also strengthens the governance of juvenile delinquency. For example, *Amendment to the Criminal Law (11)* lowers the age of criminals [8]. Wang et al. analyzed the motivation of juvenile delinquency from the perspective of juvenile delinquency psychology and theoretical basic knowledge and proposed some preventive measures for juvenile delinquency psychology [9]. Baglivio et al. studied the importance and value of juvenile delinquency correction and conducted a theoretical analysis of the psychological characteristics and core incentives of juvenile delinquency [10]. The governance of juvenile delinquency from a legal perspective will undoubtedly help strengthen external governance, but the deep-seated problem is the “internal problems” reflected in juvenile delinquency, such as the types of juvenile delinquency and the psychological characteristics of the criminal groups formed by the types. It still needs to be further explored [11]. From the point of juvenile delinquency psychology, crime prevention research can not only form a warning effect of prevention but also can timely intervene in the healthy behavior of juveniles through the construction of a criminal psychological characteristic model, to construct crime prevention at the level of juvenile's healthy behavior.

The article "Psychological Characteristics and Health Behavior for Juvenile Delinquency Groups" was retracted in 2024. Reasons: signs of a paper mill; suspected computer-generated content; unreliable results or conclusions; lack of ethics approval or compliance.

After the literature is fully analyzed and reviewed, the psychological characteristics of the juvenile delinquency groups are studied. First, the questionnaire of YPPQ is compiled according to the standard of questionnaire preparation and referring to the research results of existing literature. Then, comparing the YPPQ scores of different groups and the odds ratios (OR) values of different groups in different dimensions, the correlation between the dimensions of the scale and the interview form is analyzed, and the results of the OR values of the scales in different groups are discussed. The data is analyzed in detail through mathematical statistics, the types and characteristics of juvenile delinquency are clarified, and different criminal psychological characteristics are further excavated and classified, to construct a criminal psychological characteristic model. At last, the health behaviors of the juvenile delinquency groups are intervened in order to effectively prevent juvenile delinquency.

## 2. Research on Psychological Characteristics of Juvenile Delinquency Groups

### 2.1. Research Objects

The research objects of this study are divided into the experimental group and the control group. The research objects of the experimental group are juvenile offenders from a local juvenile detention center. In addition, the research objects of the experimental group also include adolescents with psychological problems in school psychological tests. The control group are the adolescents of the normal youth group. The number of research objects is 300. The education they receive is from primary school to junior college, and their age is around 18 years old. After the advantages of the experimental group and the control group are analyzed, the juvenile offenders are divided into the recidivism group and the nonrecidivism group.

### 2.2. Research Methods

The research test is carried out by a combination of the literature research method and questionnaire survey method. The questionnaire survey adopts the procedure of questionnaire preparation, draws on the existing research results, and compiles the YPPQ. The scale has 30 questions, and strict reliability and validity tests are carried out. The test results show that the questionnaire meets the psychometric standards [12].

The scale is used to test the psychology of the juvenile delinquency groups, in the form of written tests [13]. The scale covers rebellious society, family problems, school behavior, social cognition, legal concepts, impulsive tendencies, anger, and explicit hostility [14]. The subscales are symbolized by ANT, FAM, SCH, SOC, DQ, VIO, ANG, and HOS [15]. In addition, structured interviews are conducted to gain a more specific understanding of the psychological state of the problem youth group. The content of the interview involves 8 dimensions, including the growth environment, the family situation, impulse, antisocial, bad records, informed person evaluation, suicide, and self-evaluation [16]. Each test item is specifically operated by psychological professionals. Before the test, unified guidance is given to explain the test purpose, meaning, and requirements to the subjects. Finally, the interview results of the problem youth group are input into the computer for coding. The contents of YPPQ are exhibited in Table 1.

The article "Psychological Characteristics and Health Behavior for Juvenile Delinquency Groups" was retracted in 2024. Reasons: signs of a paper mill; suspected computer-generated content; unreliable results or conclusions; lack of ethics approval or compliance.

### 2.3. Statistical Survey

In this study, a total of 300 test questionnaires are distributed and 295 are recovered, with an effective recovery rate of 98.33%. Five invalid questionnaires are excluded, and 290 valid questionnaires are finally obtained, with an effective rate of 96.67%. The scores of the valid questionnaire are statistically analyzed, and SPSS25.0 software is used for detailed analysis. In addition, the scores of the interview and the questionnaire of the problem youth group also need descriptive statistical analysis. In this study, the reliability and validity of the YPPQ are tested by using Cronbach's *α* coefficient to test the reliability of the questionnaire [17], and it is used to test the consistency of all items or the total scale of each factor in the scale. Cronbach's *α* coefficient of the questionnaire is 0.93, and the reliability of the questionnaire is very high. For the validity of the scale [18], Kaiser-Meyer-Olkin (KMO) and Bartlett's test are used. The KMO value is between 0.9 and 1 [19], indicating that there is a strong correlation between variables, and the variables are suitable for factor analysis. The Bartlett test is significant (*p* < 0.05), and the questionnaire is highly valid. The way to test the moderating effect using SPSS software is as follows: first, the observed values of the independent and moderator variables are normalized, and the product term is constructed. The purpose of this is to reduce the multicollinearity problem among the variables in the regression equation. Then, the control variable, independent variable, moderating variable, and product term are put into the multivariate hierarchical regression model and the dependent variable in turn to test the moderating effect.

## 3. Research Results on Psychological Characteristics of Juvenile Delinquency Groups

### 3.1. Comparison of YPPQ Scores of Different Groups

The general statistical results of different groups of adolescents are shown in Figure 1.

The subjects of this study are divided into three groups: the juvenile delinquency group, the problem youth group, and the normal youth group.  Figure 1(a) shows descriptive statistics on the educational background of the three groups of subjects. Among the juvenile delinquency group, secondary school education accounted for more than 60%, followed by primary school education. The majority of the delinquency among the problem youth group are also middle school students, followed by high school students. High school students have the highest crime rate among the normal youth group, followed by middle school students.  Figure 1(b) demonstrates the ages of the three groups of research subjects, the ages are relatively similar, and the approximate age is about 18 years old. Although the age of adolescents is the closest to that of adults, their psychological states are not mature. And there are some differences between their psychological age and physiological age, which leads to insufficient understanding of themselves and easy deviant behaviors of these adolescents.

The article "Psychological Characteristics and Health Behavior for Juvenile Delinquency Groups" was retracted in 2024. Reasons: signs of a paper mill; suspected computer-generated content; unreliable results or conclusions; lack of ethics approval or compliance.

The scores of the YPPQ test of different groups and the results of the structural interview of problem youths are shown in Figure 2.

Figure 2(a) denotes the crime test scores of the three groups of research subjects in different dimension subscale items, and Figure 2(b) refers to the cause statistics of the three groups of psychological disorders for the problem youth group, including roughly eight aspects. Specifically, it covers impulsive personality problems, family environment problems, antisocial personality problems, living conditions problems, bad records problems, self-evaluation, insider evaluation, and suicide. The results of the YPPQ test signify that the juvenile delinquency group and the problem youth group have similar scores in each dimension of the scale, and the problem youth group has higher test scores in five of the dimensions than the juvenile delinquency group. And the scores of the two groups are significantly higher than that of the normal youth group, illustrating that the probability of crime is high. The normal youth group has the lowest scores in each dimension of the scale, with the lowest score of SCH and the highest score of HOS. The lower the score, the lower the probability of committing a crime. To explore the root causes of psychological disorders in the problem youth group, structured interviews are conducted in this study. The interview results show that the proportion of adolescents who have impulsive personality is close to 80%, that the proportion of adolescents who have antisocial personality problems is more than 60%, that the proportion of adolescents who have family environment problems is close to 70%, that the proportion of adolescents who have living situation problems is close to 35%, and that the proportion of adolescents who have bad records is more than 20%. The interview results are compared with the test results, and the comparison shows that this psychological test has a good effect on improving the psychological states of adolescents.

### 3.2. OR (Odds Ratio) Values of Different Groups in Different Dimensions

The OR values of different groups of adolescents and the normal youths in SCH and FAM scales are shown in Figure 3.

The article "Psychological Characteristics and Health Behavior for Juvenile Delinquency Groups" was retracted in 2024. Reasons: signs of a paper mill; suspected computer-generated content; unreliable results or conclusions; lack of ethics approval or compliance.

The juvenile delinquency group is divided into the recidivist group and the nonrecidivist group to make a more detailed analysis of the differences among the juvenile delinquency group, the problem youth group, and the normal youth group. These two groups and the problem youth group form the experimental group. The experimental group is compared with the normal youth group. The test results of the SCH and FAM scales show that the OR values of the experimental groups and the normal youth group on each question in the SCH scale are all greater than 1, which can explain the seriousness of the problems in the experimental group.

Similarly, the OR values of the FAM scale of the recidivist adolescents group, nonrecidivist adolescents group, problem youth group, and normal youth group show that the OR values on many questions are greater than 1. It cannot be ignored that the OR values of the recidivist group on question 9 are less than 1, while the OR values of the nonrecidivist group on questions 1, 5, and 9 are less than 1.

The OR values of different groups and normal group in the VIO and ANT scales are shown in Figure 4.

Figure 4(a) shows the OR values of different groups of adolescents compared with normal youths in the VIO scale. It shows that most OR values of the recidivist group, nonrecidivist group, problem youth group, and normal youth group are greater than 1 in the VIO scale. However, it is not difficult to see that the OR value of the recidivism group on question 8 is less than 1.  Figure 4(b) shows the OR values of different groups of adolescents in the ANT scale compared with normal youths. The OR values of the recidivism adolescents group, the nonrecidivism adolescent group, the problem youth group, and the normal youth group in the VIO scale are greater than 1. Similarly, the OR value of the recidivism group on question 6 is less than 1, and the OR value of the nonrecidivism group on questions 3 and 5 are less than 1.

The OR values of different groups of adolescents and normal youth in DQ and ANG scales are shown in Figure 5.

Figure 5(a) shows the OR values of different groups of adolescents in the DQ scale compared with normal youths. It can be observed that most OR values of the recidivism adolescents group, the nonrecidivism adolescents group, the problem youth group, and the normal youth group in the VIO scale are greater than 1. However, it can be found that the OR values of the recidivism group on question 3 are less than 1.  Figure 5(b) shows the OR values of different groups of adolescents compared with normal youths in the ANG scale. It can be observed that the OR values of the recidivism group, the nonrecidivism group, the problem youth group, and the normal youth group in the VIO scale are all greater than 1. Unfortunately, the OR values on all the questions in the scale are less than 1.

The article "Psychological Characteristics and Health Behavior for Juvenile Delinquency Groups" was retracted in 2024. Reasons: signs of a paper mill; suspected computer-generated content; unreliable results or conclusions; lack of ethics approval or compliance.

The OR values of different groups of adolescents and the normal youth group in the HOS and SOC scales are shown in Figure 6.

Figure 6(a) shows the OR values of different groups of adolescents compared with the normal youths in the HOS scale. It can be observed that the OR values of the recidivist adolescents group, the nonrecidivist adolescents group, the problem youth group, and the normal youth group in the VIO scale are greater than 1. There is no question whose OR value is less than 1 in the HOS and SOC scales.  Figure 6(b) shows the OR values of different groups of adolescents compared with normal youths in the SOC scale. It can be observed that most OR values of the recidivism adolescents group, the nonrecidivism adolescents group, the problem youth group, and the normal youth group in the VIO scale are greater than 1, and the OR values of the recidivism adolescents group and the non-recidivism adolescents group are less than 1.

### 3.3. Correlation between the Scale and the Interview

The results of the correlation analysis of each dimension of the scale and the interview are shown in Figure 7.

In Figure 7, SOC stands for Social Cognitive Scale, HOS refers to Overt Hostility Scale, ANG means Anger Out of Control Scale, DQ shows Legal Concept Scale, ANT indicates Antisocial Scale, VIO denotes Impulsive Tendency Scale, FAM illustrates Family Problems Scale, and SCH demonstrates School Behavior Scale. It can be seen from the correlation analysis results of each dimension of the different dimension scale and each dimension of the interview table. The correlation analysis results of each dimension of the different dimension scales and each dimension of the interview form show that the SCH scale has a significant correlation with the two questions of “bad records” and “family atmosphere” in the interview. The FAM scale is significantly correlated with the two questions of “bad records” and “impulse control” in the interview. The VIO scale, the SOC scale, and the ANT scale have no significant correlation with each dimension of the interview. The DQ scale is significantly correlated with the two questions of “impulse control” and “bad records” in the interview. The ANG scale is significantly correlated with the three questions of “family atmosphere,” “antisociety,” and “bad records” in the interview. The HOS scale is significantly correlated with the question of “impulse control” in the interview.

The article "Psychological Characteristics and Health Behavior for Juvenile Delinquency Groups" was retracted in 2024. Reasons: signs of a paper mill; suspected computer-generated content; unreliable results or conclusions; lack of ethics approval or compliance.

### 3.4. Discussion on the Results of OR Values of Different Groups in the Scales

The OR value is a commonly used indicator of epidemiology, which reflects the risk of a certain exposure factor for disease [20]. In this study, it is used to reflect the risk of test questions and measurement content for juvenile delinquency. If the OR values of most test questions in this scale are greater than 1, illustrating the content of the scale has a high correlation, and these test questions can better predict the tendency of juvenile delinquency [21]. However, there are also some test questions whose OR values are less than 1, indicating the ability of these test questions to predict juvenile delinquency needs to be further improved [22]. The test questions with fewer advantages are shown in four situations.

First, the ORs of recidivists and problem adolescents are relatively large, while those of nonrecidivists are relatively small. This may be because these test questions have the characteristics of violence or bad behavior habits. A nonrepetitive offender is usually crime of passion. They may not have long-term violent habits. Therefore, the recognition rate of these items is low or there is no significant difference from the normal group. Second, the OR values of the recidivism youth group are smaller. The reason may be that the traits measured by these questions reflect the lighter criminal tendencies. For recidivists, the recognition rate is closer to the normal group. Third, the OR values of the recidivism experimental group are high, and the recognition rate of the problem youth group is low. It could be that these tests reflect a high level of criminal tendencies, which is not suitable for young people with psychological problems. However, these problems are very necessary in psychological tests, which can effectively monitor teenagers with serious criminal tendencies. Fourth, the OR values of the three groups of crime tendency are low, which may be because the content is not suitable, and it needs to be adjusted. In general, in addition to external factors, juvenile delinquency also has some major internal factors, such as lack of self-control, the formation of a bad ego, and the influence of media and social structure, which may constitute juvenile delinquency. Therefore, society, schools, and families must play a full role in preventing crimes.

### 3.5. Analysis of the Psychological Characteristics of Juvenile Delinquency Groups

#### 3.5.1. Analysis of the Basic Characteristics of Juvenile Delinquency

Juvenile delinquency has universal physical and psychological characteristics [23]. It will be explained from the two aspects of crime subject and crime method. The details are displayed in Figure 8.

The article "Psychological Characteristics and Health Behavior for Juvenile Delinquency Groups" was retracted in 2024. Reasons: signs of a paper mill; suspected computer-generated content; unreliable results or conclusions; lack of ethics approval or compliance.

In Figure 8, from the perspective of criminal subjects, the age of crime is getting younger and younger, and the educational level is generally low. Another large proportion of juvenile delinquency appears in those who enter society prematurely. They are driven by social material desires at the school-appropriate stage, and they skip classes and drop out of school without completing their education. At the same time, adolescents are affected by various factors of information diversification, resulting in psychological and physical precocious puberty. From the perspective of the repetition of the criminal cycle, the same person has two or more criminal experiences, and the most obvious feature is a continuous crime. From the perspective of crime methods, juvenile delinquency is violent and brutal, and it is mostly manifested as intentional homicide, intentional injury, robbery, explosion, and crowd fights. The main reason is that psychology is not yet mature, and then, the irrational violent crime is carried out. More than half of the crimes belong to joint crimes, which are induced by external situations, with simple motives and prominent motives of greed.

#### 3.5.2. Analysis of Psychological Characteristic Model of Juvenile Delinquency

After sorting out, it is divided into the following psychological characteristics models of delinquency.:

1. Rebellious psychology of juvenile delinquency groups: in the growth stage, adolescents often have certain rebellious psychology [24]. Due to the “processing” of various factors such as family, school, and society, their psychology has become distorted, and eventually, they will go on the road of breaking the law and committing crimes. There are major problems in family education, and parents' long-term criticism and accusations make them form bad characters [25]. In terms of school education, teachers treat them differently according to their grades, which leads to deviations in the education method. It makes students feel pessimistic and misanthropic and develops bad characteristics such as arrogance, self-will, and impulsiveness. As for the students themselves, they are prone to give up on themselves, become depressed, and are easily influenced by the criminal subculture and embark on the road of illegality [26]
2. Weak awareness of the rule of law among juveniles: through the investigation of the social environment of juvenile delinquency, it is found that such people will do anything to resolve conflicts and lack the concept of the rule of law [27]. It is mainly affected by its growing environment, resulting in a weak legal concept. In the process of educating young people, only moral education is emphasized and the importance of legal education is ignored [28]
3. Teenagers' imitation and curiosity: juvenile delinquency groups are still at the undefined stage in their life. The juvenile delinquent group is in the unsettled stage in all aspects, easily influenced by bad culture, driven by curiosity, tendency, and imitation, which increases the probability of imitating criminal incidents [29]. In the context of the development of the Internet, teenagers' online morality has not been fully paid attention to by the family, society, and schools, resulting in the lack of online morality. The impact of Internet subculture has adverse effects on adolescents [30]. Therefore, creating a clean and green Internet environment for teenagers should become one of the directions of the healthy development of the Internet in the future
4. Teenagers' comparing psychology: because family and school education have not strengthened the guidance of students' comparison psychology, this kind of psychology has arisen among young people. Driven by it, teenagers will use illegal and criminal means to obtain the things they want [31]

By sorting out the psychological formation mechanism of the juvenile delinquent group, it is found that the psychological characteristic model is mainly composed of family and school. Families are responsible for educating teenagers. Schools are an important place for them to learn knowledge, as well as moral and legal education. Schools should focus on moral education and enhance the weight of legal education.

The article "Psychological Characteristics and Health Behavior for Juvenile Delinquency Groups" was retracted in 2024. Reasons: signs of a paper mill; suspected computer-generated content; unreliable results or conclusions; lack of ethics approval or compliance.

## 4. Intervention on Psychological Health Behavior of Juvenile Delinquency Groups

Through the above types of juvenile delinquency and the psychological characteristics, it can be found that the ultimate cause of juvenile delinquency is the behavior of adolescents, and the intervention mechanism for their behavior can help to construct a “mixed hierarchical intervention model.” Since juvenile delinquency is the result of the combined action of multiple factors, it is not realistic to unilaterally intervene in the development of the health behavior of adolescents. Therefore, the intervention of adolescent health behavior should be intervened through family, school, and society [32]. The mixed hierarchical intervention model is expressed in Figure 9.

Firstly, at the family level, parents should communicate with adolescents with a high level of empathy. Since parents and adolescents are in different age groups, there are many differences in their outlook on life, values, and world views. Consequently, to make adolescents have healthy psychology and healthy behavior, parents should act like people who have empathy with teenagers in family education, which enables parents to understand teenagers' behaviors in family education. The education developed from this is an education of communication and cooperation, which enables young people to feel that their parents communicate with them as a kind of friend and form a “virtual peer” identity with their parents. They can communicate with their parents when their hobbies need financial support, conflict with classmates, and have potential psychological comparisons, so as to avoid unhealthy behaviors driven by unhealthy psychology, and eventually embark on the road of crime.

The article "Psychological Characteristics and Health Behavior for Juvenile Delinquency Groups" was retracted in 2024. Reasons: signs of a paper mill; suspected computer-generated content; unreliable results or conclusions; lack of ethics approval or compliance.

Secondly, special education should be targeted according to the types of schools, such as special education in vocational schools or alternative schools and comprehensive schools. On the one hand, adolescents should have a sense of security in school life and learning, instead of feeling depressed. On the other hand, different types of schools should be targeted at different groups of young students with different educational methods. School education should strengthen moral education and law education, enhancing the legal concept of young students.

Finally, an overall measure conducive to the protection of adolescents should be formed by strengthening the relationship between network governance and community guidance. In terms of network governance, it is necessary to integrate the government network prevention and control office, the network technology platform, and Internet practitioners to strengthen the network ecology, forming the youth network model. In addition, the Internet access of adolescents should be limited, and the network incentives affecting youth crime should be blocked. Community guidance should be strengthened by paying visits and understanding the growth of teenagers so that the mental health of teenagers can be known about and their subhealth behavior can be corrected timely.

In short, the construction of family, school, society, and other multilevel mixed intervention models can predict the psychological health of adolescents and correct their healthy behavior timely. It also promotes and protects the psychological health of adolescents through prevention and treatment and provides the targeted intervention measure of health behavior of adolescents.

## 5. Conclusion

The objectives are to pay attention to the mental health of juveniles, study the psychological characteristics of juvenile delinquency groups, implement their psychological characteristics model on this basis, then propose healthy behavior intervention strategies, and finally effectively help juvenile delinquency groups to improve their mental health problems, so as to achieve the purpose of preventing juvenile delinquency. On the basis of literature analysis, this research firstly compiled the YPPQ, and the structured interview content of the problem youth group was set up. Secondly, the questionnaire results and the interview results were unified for data processing, the correlation was studied, and the psychological characteristics model of juvenile offenders was constructed. Finally, the intervention strategy of healthy behavior was proposed. The survey results manifest that the psychological characteristics of juvenile delinquency groups are rebellious and have weak awareness of the rule of law, imitation, curiosity, and comparison. These are all momentous factors that induce juvenile delinquency. The “mixed hierarchical intervention model” is further proposed, which should focus on multilevel, multiangle, and focused interventions on adolescents' health behaviors through families, schools, and society. There are still some deficiencies. Due to the influence of objective factors, the number of research objects is limited, and the generality of the data needs to be strengthened. The development direction of future research is to continue to improve the questionnaire scale, so as to study the psychological characteristics of juvenile delinquency more generally and accurately. The advantage of this research lies in that on the basis of predecessors, the YPPQ was compiled to quantitatively analyze the psychological characteristics of juvenile delinquency from different dimensions and further propose the intervention model of healthy behavior.

The article "Psychological Characteristics and Health Behavior for Juvenile Delinquency Groups" was retracted in 2024. Reasons: signs of a paper mill; suspected computer-generated content; unreliable results or conclusions; lack of ethics approval or compliance.

## Figures and Tables

**Figure 1:** General statistics of different groups of adolescents ((a) education and (b) age).

**Figure 2:** Scores of the YPPQ test of different groups of adolescents and the interview on problem youths ((a) YPPQ test and (b) structural interview results of problem youths).

**Figure 3:** OR values of different groups of adolescents compared with normal youths in SCH and FAM scales ((a) OR values in SCH scale and (b) OR values in FAM scale).

**Figure 4:** OR values of different groups of adolescents in VIO and ANT scales compared with normal youths ((a) OR values in VIO scale and (b) OR values in ANT scale).

**Figure 5:** OR values of different groups of adolescents in DQ and ANG scales compared with normal youths ((a) OR value in the DQ scale) and (b) OR value in the ANG scale).

**Figure 6:** OR values of different groups of adolescents compared with normal youths in the HOS and SOC scales ((a) OR values in the HOS scale and (b) OR values in the SOC scale).

**Figure 7:** Results of correlation analysis of the scale and the interview.

The article "Psychological Characteristics and Health Behavior for Juvenile Delinquency Groups" was retracted in 2024. Reasons: signs of a paper mill; suspected computer-generated content; unreliable results or conclusions; lack of ethics approval or compliance.

**Figure 8:** Basic characteristics of juvenile delinquency.

**Figure 9:** The mixed hierarchical intervention model.

**Table 1:** The contents of YPPQ.

No.	Contents covered	Abbreviation for subscale
1	Antisocial	ANT
2	Family issues	FAM
3	School behavior	SCH
4	Social cognition	SOC
5	Legal concept	DQ
6	Impulsive tendencies	VIO
7	Anger out of control	ANG
8	Overt hostility	HOS

## Data Availability

The data used to support the findings of this study are included within the article.
